The article "Effects of Task-Based LSVT-BIG Intervention on Hand Function, Activity of Daily Living, Psychological Function, and Quality of Life in Parkinson's Disease: A Randomized Control Trial" was published in 2022. Journal: Occup Ther Int.

# Effects of Task-Based LSVT-BIG Intervention on Hand Function, Activity of Daily Living, Psychological Function, and Quality of Life in Parkinson's Disease: A Randomized Control Trial

**DOI:** 10.1155/2022/1700306

**Published:** 2022-09-10

**Authors:** YoungSeok Choi, DeokJu Kim

**Affiliations:** ^1^Department of Occupational Therapy, Cheongju Samsung Hospital, Cheongju, Republic of Korea; ^2^Department of Occupational Therapy, College of Health & Medical Sciences, Cheongju University, Cheongju, Republic of Korea; ^3^Department of Occupational Therapy, Cheongju University, Daesung-ro, 298, Cheongwon-gu, Cheongju-si, Chungcheongbuk-do, Republic of Korea

## Abstract

Previous studies have demonstrated that the Lee Silverman Voice Treatment-BIG (LSVT-BIG) program can improve motor functions such as balance and gait in Parkinson's disease (PD) patients. However, no study has investigated the effects of a task-based LSVT-BIG intervention on hand function, psychological function, and quality of life in PD patients. Herein, we investigate the effects of a task-based LSVT-BIG intervention, which reflects the needs of PD patients, on hand function, activity of daily living (ADL), psychological function, and quality of life. A total of 14 PD patients were enrolled and randomly assigned to the experimental or control group. The experimental group performed 30 minutes of conventional occupational therapy and 40 minutes of the task-based LSVT-BIG program. The control group performed 30 minutes of conventional occupational therapy and 40 minutes of relaxation and stretching. Both groups underwent the respective interventions once a day 5 times a week for 4 weeks. As a result of the study, the experimental group showed improvement in hand function in both the dominant and nondominant hand, and the control group showed improvement only in the nondominant hand (*p* < .05). ADL was significantly improved in both groups, but the experimental group showed a more statistically significant difference than the control group (*p* < .05). Depression and anxiety were significantly decreased in both the experimental group and the control group, and in particular, in the case of anxiety, there was a more statistically significant difference in the experimental group (*p* < .05). In the case of the experimental group, there was a significant improvement in quality of life in all items, and in the control group, except for the social function item (*p* > .05), there was a significant improvement in other items (*p* < .05). The results of this study suggest that the task-based LSVT-BIG program, which consists of activities desired by the participants, may be an effective intervention to improve hand function, ADL, psychological function, and quality of life in PD patients.

The article "Effects of Task-Based LSVT-BIG Intervention on Hand Function, Activity of Daily Living, Psychological Function, and Quality of Life in Parkinson's Disease: A Randomized Control Trial" was published in 2022. Journal: Occup Ther Int.

## 1. Introduction

The increase in life expectancy in recent decades has led to a rapid expansion of the elderly population worldwide. This has been followed by an increase in the number of patients with chronic diseases [1]. Along with Alzheimer's disease, Parkinson's disease (PD) is a representative neurodegenerative disease. The prevalence of PD is increasing worldwide as the elderly population continues to grow [2]. PD is caused by a deficiency of dopamine, a neurotransmitter found in the substantia nigra of the brain [3]. The lack of dopamine causes abnormalities in the striatum and abnormal functions of the basal ganglia, which is controlled by the striatum [4]. Subsequently, this commonly leads to movement disorders as well as various cognitive function and emotional control disorders [5, 6]. Common movement disorders caused by the lack of dopamine include slow movement, gait disturbance, tremor, muscle stiffness, and postural instability. This limits fine movements and motions, thereby leading to difficulties in maintaining normal activity of daily living (ADL) [7]. Furthermore, bradykinesia reduces the speed, range, width, and initiation of movement. This leads to delays in reaction and movement time for buttoning, writing, eating, bathing, and dressing [3], restricting independent ADL and social participation [8].

In addition to movement disorders, cognitive impairment, mood disorders, emotional disorders, and sleep disorders can all occur in PD patients. In particular, depression is commonly observed [9] in approximately 40-70% of patients with PD [9, 10]. The number of patients with multiple psychiatric symptoms such as depression and anxiety is continuously increasing, and in about 41% of patients, depression and anxiety are observed simultaneously [11]. PD patients experience fear of losing control over their daily life due to movement disorders such as tremor, postural instability, and gait disturbance. Abnormal symptoms may lead to a feeling of social isolation, leading to subsequent anxiety [12]. These symptoms negatively affect PD patients and eventually decrease their quality of life [13].

Although PD currently has no known cure, various therapeutic approaches have been attempted to suppress disease progression and alleviate symptoms [14]. In general, pharmacological and nonpharmacological interventions are both applied as interventions. Pharmacological intervention supplements dopamine to alleviate symptoms or prevent/delay the destruction of nerve cells [15]. Long-term use of pharmacological intervention is associated with side effects such as hallucinations, delusions, insomnia, and resistance against the used regimen [16]. Nonpharmacological interventions include exercise. In fact, prior studies have shown that moderate intensity exercise can improve the function and levels of dopamine in PD patients [17]. However, there is a lack of interest in the disease in Korea, and only a limited number of clinical studies have evaluated the effects of exercise therapy for PD in Korea [18]. As the number of patients with PD is expected to increase as the population ages, it is necessary to provide treatments with proven effects to PD patients in Korea.

The article "Effects of Task-Based LSVT-BIG Intervention on Hand Function, Activity of Daily Living, Psychological Function, and Quality of Life in Parkinson's Disease: A Randomized Control Trial" was published in 2022. Journal: Occup Ther Int.

Task-based training is widely used in the rehabilitation of patients with neurological impairment. This intervention provides task-specific strategies through which the patients can practice the necessary abilities to achieve the goal of a given task and thereby improve adaptability and develop problem-solving and reward strategies [19]. Marjorie [20] showed that purposeful tasks can generate more interest than mechanically repetitive exercises, and functional tasks with real tools that improve ADL can not only motivate the patients but also improve their sense of achievement and satisfaction compared to the repeated practice of normal patterns [21–23].

The Lee Silverman Voice Treatment-BIG (LSVT-BIG) program is an intervention program for patients with PD. The LSVT-BIG was developed in 2005 based on the previous Lee Silverman Voice Treatment-LOUD program for increasing voice volume. The program is aimed at facilitating brain reconstruction and rebalancing the sensory system through high-amplitude movements. By performing standardized large movements, the program improves motion amplitude and accuracy and induces rapid movements [24]. The LSVT-BIG program includes stretching and stepping exercises, as well as activities related to ADL [25]. The therapist provides tactile and visual cues through modeling, and the intervention improves movement patterns by forming techniques, correcting senses, and improving self-awareness [26]. According to previous studies, the LSVT-BIG program is effective in improving balance and gait [14, 27, 28].

As previously described, task-based training is effective in patients with neurological impairment; however, task-based training has only been applied to patients with PD in a limited number of studies in Korea. In addition, although the LSVT-BIG program is effective for patients with PD, most studies on the LSVT-BIG program have focused on changes in physical functions, such as gait and balance. PD is a chronic disease with a prolonged disease period associated with decreased physical function and negative psychological symptoms, such as depression and anxiety and emotional atrophy. However, only a few studies have evaluated the changes in psychological symptoms. Furthermore, the LSVT-BIG program mainly consists of stretching and stepping exercises along with simple functional tasks, which show limitations in engaging patients in the activities.

The article "Effects of Task-Based LSVT-BIG Intervention on Hand Function, Activity of Daily Living, Psychological Function, and Quality of Life in Parkinson's Disease: A Randomized Control Trial" was published in 2022. Journal: Occup Ther Int.

Therefore, in this study, a task-based LSVT-BIG program using actual tools was implemented. The activities were selected based on the needs of the patients, and the effects of the task-based LSVT-BIG program on hand function, ADL, emotional state such as anxiety and depression, and quality of life were assessed.

## 2. Methods

### 2.1. Participants

This study was conducted from July to October 2021 on 14 patients with PD who were undergoing rehabilitation treatment at the S and W hospitals in Cheongju. The participant selection criteria were as follows: (1) diagnosis of PD by a specialist, (2) disease onset more than 6 months prior, (3) lack of aphasia or limitations of sight or hearing, (4) levels 1-3 on the Hoehn and Yahr scale, and (5) score of 21 points or higher on the Berg Balance Scale (BBS). The exclusion criteria were as follows: (1) history of other neurological disease, (2) difficulty participating in training due to orthopedic diseases, and (3) participation in other rehabilitation studies or drug experiments in the prior 6 months.

### 2.2. Procedure

This was a randomized controlled experimental study using a simple randomization method. The selected participants were numbered from 1 to 14 and were randomly selected to be assigned to the experimental or control group. The participants were blinded for their group assignment. This study was approved by the Institutional Review Board (IRB) of Cheongju University (1041107-202106-HR-018-01). Before recruiting the participants for the study, the sample size was calculated based on the primary outcome measure in G-Power. The effect size was set to 0.5, the significance level was set to 0.05, and the power was 80%. For enrollment, the participants underwent Hoehn and Yahr staging. Based on the results of this assessment, those who satisfied the participant selection criteria were enrolled. However, several participants could not participate in this study due to fatigue or medical problems. As a result, 14 participants were included in the final analysis. After the final selection, the participants were randomly assigned to the experimental or control group. Prior to the intervention, the experimental group completed the Canadian Occupational Performance Measure (COPM) and was instructed to self-select meaningful tasks involving upper extremity movement. The experimental group performed 40 minutes of the task-based LSVT-BIG program and 30 minutes of conventional occupational therapy in the treatment room 5 times a week for 4 weeks. Conversely, the control group performed 30 minutes of conventional occupational treatment and 40 minutes of relaxation training and stretching 5 times a week for 4 weeks. The procedure of this study is shown in Figure 1.

The article "Effects of Task-Based LSVT-BIG Intervention on Hand Function, Activity of Daily Living, Psychological Function, and Quality of Life in Parkinson's Disease: A Randomized Control Trial" was published in 2022. Journal: Occup Ther Int.

### 2.3. Outcome Measurements

The Hoehn and Yahr scale used in this study to screen PD patients is a five-stage scale developed by [29]. This tool evaluates the clinical symptoms of PD: stage 1 “unilateral tremor or stiffness at rest,” stage 2 “bilateral tremor or stiffness at rest,” stage 3 “bilateral symptoms and postural instability,” stage 4 “able to walk or stand to some extent with difficulties in independent daily life,” and stage 5 “difficulties in walking or standing and unable to lead an independent daily life” [30].

The Canadian Occupational Performance Measure (COPM) is a semistructured evaluation tool developed by Law et al. [31]. Evaluation was conducted through interviews by a therapist with the patient or caregiver. The participants evaluated whether they experienced problems in self-management, productive activities, and leisure activities on a 10-point scale (10 points = very important). The top five tasks were then prioritized to set the intervention goal. Each of the selected goals was assigned performance and satisfaction scores using a 10-point scale (10 points = very well performed, very satisfied). The performance and satisfaction scores of the selected tasks were combined and divided by the number of tasks to calculate the mean score. The test-retest reliability and internal validity of COPM are 0.84–0.92 and 0.56–0.71, respectively [32]. In this study, COPM evaluation was conducted before the experiment to select a goal for the task desired by the participant.

The Nine-Hole Pegboard, a tool to measure hand agility, was used in this study to evaluate hand agility and upper extremity motor function. The time required to insert nine pegs into the holes of the board and to subsequently pull the pegs out of the holes was measured. A shorter time indicated better hand agility. The interrater reliability of the tool is 0.98 for the right hand and 0.99 for the left hand [33].

The New ADL Questionnaire is a daily activity assessment tool developed by Lee et al. [34] focusing on the clinical symptoms of PD patients. The tool consists of 20 items such as walking in daily life, sitting on the floor and standing, taking the first step, crossing the street, climbing the stairs, using the bathroom, and taking a bath. Each item is evaluated on a 6-point scale: 0 point indicates “independent performance”; 1 point, “slow independent performance”; 2 points, “mild difficulties, but does not require help or assistance from others”; 3 points, “requires aid from a caregiver or assistive tools for less than half of the activity”; 4 points, “requires aid from a caregiver or assistive tools for more than half of the activity”; and 5 points, “requires complete help.” A lower score indicates greater independence in ADL, and the test-retest reliability of the tool is 0.79 [34].

The article "Effects of Task-Based LSVT-BIG Intervention on Hand Function, Activity of Daily Living, Psychological Function, and Quality of Life in Parkinson's Disease: A Randomized Control Trial" was published in 2022. Journal: Occup Ther Int.

The Beck Depression Inventory (BDI), a self-administered depression scale developed by Beck et al. [35], was used in this study to evaluate depression. This test consists of 21 items evaluating the patients' emotional, cognitive, motivational, physical, and other symptoms. Each item is evaluated on a 4-point scale from 0 to 3 points, and the total score can range between 0 and 63 points. A score of 0-9, 10-15, 16-23, and > 24 indicates “no depression,” “mild depression,” “moderate depression,” and “severe depression,” respectively. The reliability of the tool is 0.88 [36].

To evaluate anxiety, the State-Trait Anxiety Inventory Korean YZ (STAI-KYZ), developed by Spielberger [37] and modified to Korean by Han et al. [38], was used. The STAI-KYZ evaluates state anxiety that changes over time and trait anxiety observed in motivational or behavioral tendencies. State anxiety evaluates the emotional state of an individual “at the moment” and indicates the subjective states of agitation, tension, worry, and concern caused by activation or excitability of the autonomic nervous system. Trait anxiety evaluates the emotional state of how an individual feels “in general” and indicates anxiety at the level of an individual's innate temperament or personality that remains relatively unchanged. A total of 20 self-administered items on state and trait anxiety are evaluated on a 4-point scale: 1 point, “strongly disagree”; 2 points, “disagree”; 3 points, “agree”; and 4 points, “strongly agree.” The total score ranges from 20 to 80 points, and a higher score indicates greater anxiety. The reliability of the internal consistency of the tool is 0.89 for state anxiety and 0.88 for trait anxiety [39].

The PD quality of life questionnaire (PDQL) was used to evaluate quality of life in this study. The PDQL was developed by De Boer et al. [40] and consists of 37 self-administered items. The questionnaire consists of subdomains on PD symptoms, systemic symptoms, social function, and emotional function. Each item is evaluated on a 5-point scale from 1 to 5 points: 1 point indicates “always”; 2 points, “mostly”; 3 points, “occasionally”; 4 points, “sometimes”; and 5 points, “not at all.” A higher score indicates lower quality of life, and the reliability of the tool is 0.97 [41].

The article "Effects of Task-Based LSVT-BIG Intervention on Hand Function, Activity of Daily Living, Psychological Function, and Quality of Life in Parkinson's Disease: A Randomized Control Trial" was published in 2022. Journal: Occup Ther Int.

### 2.4. Intervention

The task-based LSVT-BIG program provided to the experimental group consisted of 15 minutes of maximal daily exercise (7 repetitive exercises), followed by 10 minutes of functional component tasks (5 types of repetitive movement training), 10 minutes of hierarchy tasks (hierarchical task performance training), and 5 minutes of BIG walking (walking in big movements). The program was reorganized based on the LSVT-BIG program standardized protocol [42] to include task-based training. Prior to the intervention, the participants completed the COPM to self-select meaningful tasks. The selected tasks were applied to the functional components and hierarchy tasks (Tables 1 and 2 and Figures 2(a)–2(c)). The relaxation and stretching program completed by the control group was developed to stabilize negative emotions and maintain and improve physical functions. The progressive muscle relaxation technique [43], in which the participant intentionally contracts and relaxes muscles to find psychological stability, was reconstructed to allow both the mind and body to relax with meditation. Stretching improves muscle strength through repeated contraction and extension of muscles. In this study, the stretching exercises for the elderly presented by Kim [44] were replicated according to the conditions of the participants. The stretching exercises included activities such as bending the trunk, straightening the chest, turning the trunk left and right, and lifting the shoulders.

### 2.5. Statistical Analysis

SPSS version 24.0 was used for all statistical analysis in this study. The Shapiro-Wilk test was conducted to test the normality of the data. As normality was not met, nonparametric analysis was conducted. Chi-square test and descriptive statistics were conducted for the general characteristics of the participants. The Mann-Whitney *U* test was conducted to test functional homogeneity before intervention. The Wilcoxon signed rank test was performed to compare the pre- and postintervention intragroup differences of the two groups, and the Mann-Whitney *U* test was conducted to compare pre- and postintervention differences between the groups. The statistical significance level of all data was set to 0.05.

## 3. Results

### 3.1. General Characteristics of the Research Subjects

The general characteristics of the participants are as follows (Table 3). The experimental group consisted of six men (85.71%) and one woman (14.29%). In the control group, three men (42.86%) and four women (57.14%) were included. The mean age was 71.57 ± 7.74 and 70.86 ± 8.49 years in the experimental and control groups, respectively. The BBS score was 39.86 ± 2.60 and 40.00 ± 4.04 points, and the Hoehn and Yahr score was 2.43 ± 0.53 and 1.85 ± 0.69 points in the experimental and control groups, respectively. There were no significant differences in age, sex, BBS score, or Hoehn and Yahr levels between the two groups (*p* > .05).

The article "Effects of Task-Based LSVT-BIG Intervention on Hand Function, Activity of Daily Living, Psychological Function, and Quality of Life in Parkinson's Disease: A Randomized Control Trial" was published in 2022. Journal: Occup Ther Int.

### 3.2. Comparison of Hand Function before and after Intervention

The Nine-Hole Pegboard Test was conducted to evaluate the before and after intervention hand function of the two groups. In the experimental group, the score for the dominant hand decreased from 26.63 ± 10.25 points before intervention to 22.57 ± 8.63 points after intervention, and the score for the nondominant hand decreased from 42.59 ± 37.68 points before intervention to 30.69 ± 22.41 points after intervention. Both hands showed significant changes in function (*p* < .05). In the control group, the dominant hand showed no significant change. However, the score for the nondominant hand decreased significantly from 32.87 ± 24.54 points before intervention to 30.24 ± 22.09 points after intervention (*p* < .05). The change in the nondominant hand was significantly different between the two groups (*p* < .05) (Table 4).

### 3.3. Changes in Activity of Activity of Daily Living before and after Intervention

The changes in ADL before and after intervention were assessed. In the experimental group, the ADL score decreased significantly from 36.28 ± 21.80 points before intervention to 27.71 ± 19.02 points after intervention (*p* < .05). Similarly, in the control group, the ADL score decreased significantly from 36.14 ± 11.92 points before intervention to 33.57 ± 11.58 points after intervention (*p* < .05). However, the change in ADL score after intervention was significantly different between the two groups (*p* < .05) (Table 5).

### 3.4. Changes in Psychological Function after Intervention

The changes in BDI before and after intervention were assessed. In the experimental group, BDI score decreased significantly from 46.14 ± 11.33 points before intervention to 38.85 ± 11.46 points after intervention (*p* < .05). Similarly, in the control group, the BDI score decreased significantly from 43.00 ± 7.54 points before intervention to 39.57 ± 7.52 points after intervention (*p* < .05). However, the change in depression was not significant between the two groups (*p* > .05). Changes in STAI-KYZ after intervention were evaluated in both the experimental and control groups. In the experimental group, the state anxiety score decreased significantly from 56.71 ± 9.01 points before intervention to 45.42 ± 8.34 points after intervention, while the trait anxiety score similarly decreased significantly from 57.42 ± 10.37 to 49.71 ± 10.33 points (*p* < .05). In the control group, state anxiety score decreased significantly from 51.14 ± 10.23 to 45.85 ± 9.02 points (*p* < .05), and the trait anxiety score decreased significantly from 48.71 ± 6.84 points before intervention to 46.28 ± 6.47 points after intervention (*p* < .05). The changes in state and trait anxiety score were significantly different between the two groups (*p* < .05) (Table 6).

The article "Effects of Task-Based LSVT-BIG Intervention on Hand Function, Activity of Daily Living, Psychological Function, and Quality of Life in Parkinson's Disease: A Randomized Control Trial" was published in 2022. Journal: Occup Ther Int.

### 3.5. Changes in Quality of Life before and after Intervention

The changes in quality of life after intervention in the two groups can be summarized as follows (Table 7). In the experimental group, the subdomain and total score were significantly changed (*p* < .05). In contrast, the control group showed significant changes in the scores of all items (*p* < .05), excluding social function (*p* > .05). There were no significant differences in changes in quality of life between the two groups (*p* > .05).

## 4. Discussion

In this study, we evaluated the effects of implementation of the task-based LSVT-BIG program on hand function, ADL, mental health, and quality of life in PD patients. Compared to previous LSVT-BIG programs which included functional task training and hierarchical task training focused on movements using large muscles, the task-based LSVT-BIG program applied in this study consisted of task-based training using real tools and large movements involving large muscles. Prior to selecting the tasks, the participants completed the COPM and were consulted by therapists to select three hierarchical tasks that could increase participation motivation. Each of these hierarchical tasks was divided into three stages, and the program was structured to include large movements of the upper and lower limbs and movement of the hand that manipulated objects step by step. Functional task training consisted of five functional movements that could help perform hierarchical tasks. Before starting a hierarchical task, five related functional tasks were first practiced.

The results of the Nine-Hole Pegboard Test showed that the function of both the dominant and nondominant hands decreased after intervention in the experimental group. Conversely, in the control group, only the nondominant hand showed significant changes after intervention. The experimental group showed a more significant difference in the function of the nondominant hand. The task-based LSVT-BIG program included various activities that required hand movement, such as moving or manipulating an object. The experimental group efficiently performed the desired tasks in a familiar treatment environment, which would have contributed to the observed improved agility of the hands. Consistent with our findings, Kim et al. [45] showed that task-based training consisting of tasks mainly used in daily life improved the upper extremity function and balance in stroke patients. Additionally, Noh et al. [46] observed that tasks of ADL, including grabbing objects, picking, controlling, manipulating, and using muscle strength, enhanced hand function (manipulative ability), further supporting our findings.

The article "Effects of Task-Based LSVT-BIG Intervention on Hand Function, Activity of Daily Living, Psychological Function, and Quality of Life in Parkinson's Disease: A Randomized Control Trial" was published in 2022. Journal: Occup Ther Int.

After the intervention, ADL was significantly improved in both groups; however, the increase was significantly greater in the experimental group than in the control group. The change in ADL score was significantly different between the two groups. Although the respective interventions of the experimental and control groups had positive effects on ADL, the intervention involving meaningful daily activity tasks selected by the participants themselves was more effective at enhancing daily activity performance levels. Bloem et al. [47] reported that postural instability, which is one of the characteristics of PD patients, was the biggest cause of falls and that falls from postural instability increased fear of ADL. The task-based LSVT-BIG program provided to the experimental group included not only repetitive movements such as extending arms and stepping back and forth but also functional tasks that are frequently used in daily life and hierarchical tasks requiring complex movement control. These activities are thought to have improved movement planning, control, and body coordination. This subsequently led to ameliorated postural stability and balance, improving the ADL score.

In this study, depression and anxiety were evaluated to investigate the psychological function of PD patients, and depression was found to be significantly reduced in both the groups. If depressed mood persists, participation in daily physical activities such as eating, sleeping, and personal hygiene decreases, leading to functional impairment. As a result, depression is aggravated, and this vicious cycle is repeated. Hotting and Roder [48] reported that regular and adequate intensity exercise improves cognitive functions such as memory, concentration, and executive function and positively affects emotions by relaxing and stabilizing the mood, highlighting the importance of exercise. In our study, both the experimental and the control group underwent regular moderate-intensity exercises involving muscle relaxation therapy and stretching. This seems to have improved emotional stability, decreasing the severity of depression in PD patients.

Both state and trait anxiety decreased in the experimental and control groups. However, the decrease was more significant in the experimental group than in the control group. State anxiety shows the “current” emotional state of an individual and evaluates agitation, tension, and concern caused by the activation or excitement of the autonomic nervous system. Trait anxiety refers to one's “general” emotional state and is a measure of anxiety at rest. Restriction of body functions leads to a reduction in ADL. This, in turn, causes changes in personality, behavior, and mindset [49]. The experimental group repeatedly finished conducting tasks of various functional activities. This improved the patients' emotional stability, changed their mindset, and subsequently alleviated both state and trait anxiety. The experimental group showed a more significant decrease in anxiety than the control group, indicating that the LSVT-BIG program may be a useful method to prevent anxiety in patients with PD.

The article "Effects of Task-Based LSVT-BIG Intervention on Hand Function, Activity of Daily Living, Psychological Function, and Quality of Life in Parkinson's Disease: A Randomized Control Trial" was published in 2022. Journal: Occup Ther Int.

Herein, we assessed the changes in the quality of life of both the experimental and control groups. In the experimental group, positive changes in the subdomain and total scores of quality of life were observed. Conversely, the control group showed no significant changes in social function. The task-based LSVT-BIG program consists of daily life movements which reflect the individual needs of the patients. This provides strong motivation to complete the tasks [50], thereby improving the upper extremity function and emotions such as anxiety and depression. As a result, this would have improved the quality of life. Unlike the experimental group, which showed significant changes in all subdomains of quality of life, the control group showed no significant change in social function. Physical disorders in PD patients increase dependence of the patients on others for daily activities and promote reluctance for social participation [51]. In our study, the experimental group showed increased confidence in social participation through repeating training of daily activities with motivation. In contrast, although the progressive muscle relaxation therapy and stretching performed by the control group positively increased the quality of life related to symptoms of PD, systemic symptoms, and emotional function, the program may have lacked the motivation to provoke social participation, leading to differences in the improvement of social function between the two groups.

The findings of this study showed that the task-based LSVT-BIG program positively affected upper extremity function, depression, anxiety, and quality of life in PD patients. However, several limitations must be considered in the interpretation of this study's findings. First, only a small number of participants were included in this study, and therefore, the findings cannot be generalized for all PD patients. Second, it is thought that improved balance leads to increased hand function and ADL; however, the changes in balance after intervention were not directly evaluated. Lastly, the intervention period was short at only 4 weeks, and the lack of follow-up means it is unclear whether the effects of the program persisted in the long term. Therefore, follow-up studies must be conducted on a large number of participants to select tests that can prove the various effects of the program. Additionally, it would be necessary to determine the continuity of the effects of the task-based LSVT-BIG intervention.

The article "Effects of Task-Based LSVT-BIG Intervention on Hand Function, Activity of Daily Living, Psychological Function, and Quality of Life in Parkinson's Disease: A Randomized Control Trial" was published in 2022. Journal: Occup Ther Int.

## 5. Conclusion

We constructed a task-based LSVT-BIG program consisting of activities meaningful to the PD patients. We found that application of this program significantly improved the hand function, ADL, mental health, and quality of life of PD patients. Thus, our findings suggest that a task-based LSVT-BIG program may be an effective intervention method for patients with PD.

## Figures and Tables

**Figure 1:** Flow chart. COPM: Canadian Occupational Performance Measure; BDI: Beck Depression Inventory; STAI-KYZ: State Trait Anxiety Inventory-Korean; PDQL: Parkinson's Disease Quality of Life Questionnaire. ^∗^COPM was conducted only in the experimental group.

**Figure 2:** Functional component tasks and hierarchy tasks reflecting the tasks performed by participants with images (example of participant A).

**Table 1:** Description of the Lee Silverman Voice Treatment-BIG (original protocol).

Stage	Time	Intervention
Maximal daily exercise	15 minutes	(1) Stretching the arm to reach the ceiling from the floor, 8 reps (2) Extending the arm from side to side, 8 reps (3) Stepping forward, 8 reps (4) Stepping sideways, 8 reps (5) Steeping backwards, 8 reps (6) Extending the arm by shaking forward and backward, 10 reps (7) Stepping sideways while turning the torso, 10 reps

Functional component tasks	10 minutes	5 functional movement tasks (5 reps)

Hierarchy tasks	10 minutes	1–3 hierarchical tasks

BIG walking	5 minutes	Walking with big movements

**Table 2:** Functional component tasks and hierarchy tasks reflecting the needs of participants (example of participant A).

COPM goal	Functional component tasks	Hierarchy tasks
Bathing	(i) Walking in big motions (ii) Throwing and receiving a ball (iii) Touching the head, shoulders, knees, and feet with both hands in a standing position (iv) Touching the back of the head, back, buttocks, and heels with both hands in a standing position (iv) Rotating both arms	(i) Motion of holding a towel and applying soap on the body (ii) Motion of rinsing the body with water and hands (iii) Motion of wiping the body with a towel

Cleaning	(i) Sitting and standing up from a chair (ii) Walking in big motions (iii) Rotating the body with arms outstretched in a standing position (iv) Extending the arms in multiple directions (v) Folding the towel into three even parts	(i) Getting up and walking to pick up a towel (ii) Cleaning the desk with a towel (iii) Folding the used towel, putting it in a basket, and returning to a chair

Bowling	(i) Walking in big motions (ii) Throwing a ball with one hand in a standing position (iii) Extending the arms in multiple directions in a standing position (iv) Bending the back to touch the ground in a standing position (v) Placing bowling pins upright on the ground	(i) Getting up from a chair and walking to grab a bowling ball (ii) Striking down bowling pins with a bowling ball (iii) Reorganizing bowling pins upright and returning back to a chair to sit

The article "Effects of Task-Based LSVT-BIG Intervention on Hand Function, Activity of Daily Living, Psychological Function, and Quality of Life in Parkinson's Disease: A Randomized Control Trial" was published in 2022. Journal: Occup Ther Int.

**Table 3:** General characteristics of the subjects (*N* = 14).

	EG (*n* = 7)		CG (*n* = 7)		*p*
Age (years)	71.57 ± 7.74^†^		70.86 ± 8.49		.798
Sex (*n* (%))					
Male	6	85.71	3	42.86	.107
Female	1	14.29	4	57.14	
BBS (score)	39.86 ± 2.60		40.00 ± 4.04		.694
H&Y (score)	2.43 ± 0.53		1.85 ± 0.69		.114

^†^Mean ± SD. ^∗^*p* < .05. BBS: Berg Balance Scale; H&Y: Hoehn-Yahr Scale; EG: experimental group; CG: control group.

**Table 4:** Changes of Nine-Hole Pegboard Test before and after intervention (*N* = 14).

			Pretest	Posttest	*Z*	*p*	Difference	*Z*	*p*
9-Hole	EG	Dominant hand	26.63 ± 10.25^†^	22.57 ± 8.63	-2.366	.018^∗^	−4.06 ± 1.62	-1.086	.277
	CG		27.02 ± 20.32	24.78 ± 17.65	-1.521	.128	−2.24 ± 2.67		
	EG	Nondominant hand	42.59 ± 37.68	30.69 ± 22.41	-2.366	.018^∗^	−11.90 ± 15.27	-2.364	.018^∗^
	CG		32.87 ± 24.54	30.24 ± 22.09	-2.366	.018^∗^	−2.63 ± 2.45		

^†^Mean ± SD. ^∗^*p* < .05. 9-Hole: Nine-Hole Pegboard Test; EG: experimental group; CG: control group.

**Table 5:** Changes of the New ADL Questionnaire before and after intervention (*N* = 14).

	Pretest	Posttest	*Z*	*p*	Difference	*Z*	*p*
ADL-Q							
EG	36.28 ± 21.80^†^	27.71 ± 19.02	-2.201	.028^∗^	−8.57 ± 2.78	-2.187	.029^∗^
CG	36.14 ± 11.92	33.57 ± 11.58	-2.226	.026^∗^	−2.57 ± 0.34		

^†^Mean ± SD. ^∗^*p* < .05. ADL-Q: the New ADL Questionnaire; EG: experimental group; CG: control group.

**Table 6:** Changes of psychological function before and after intervention (*N* = 14).

	Pretest	Posttest	*Z*	*p*	Difference	*Z*	*p*
BDI							
EG	46.14 ± 11.33^†^	38.85 ± 11.46	-2.366	.018^∗^	−7.29 ± 0.13	-1.355	.175
CG	43.00 ± 7.54	39.57 ± 7.52	-2.376	.017^∗^	−3.43 ± 0.02		
STAI-KYZ(S)							
EG	56.71 ± 9.01	45.42 ± 8.34	-2.375	.018^∗^	−11.29 ± 0.67	-2.374	.018^∗^
CG	51.14 ± 10.23	45.85 ± 9.02	-2.375	.018^∗^	−5.29 ± 1.21		
STAI-KYZ(T)							
EG	57.42 ± 10.37	49.71 ± 10.33	-2.384	.017^∗^	−7.71 ± 0.04	-2.132	.033^∗^
CG	48.71 ± 6.84	46.28 ± 6.47	-2.207	.027^∗^	−2.43 ± 0.37		

^†^Mean ± SD. ^∗^*p* < .05. BDI: Beck Depression Inventory; STAI-KYZ(S): State Trait Anxiety Inventory-Korean YZ-state anxiety; STAI-KYZ(T): State Trait Anxiety Inventory-Korean YZ-trait anxiety; EG: experimental group; CG: control group.

The article "Effects of Task-Based LSVT-BIG Intervention on Hand Function, Activity of Daily Living, Psychological Function, and Quality of Life in Parkinson's Disease: A Randomized Control Trial" was published in 2022. Journal: Occup Ther Int.

**Table 7:** Changes of state Parkinson's Disease Quality of Life Questionnaire before and after intervention (*N* = 14).

	Pretest	Posttest	*Z*	*p*	Difference	*Z*	*p*
Parkinsonian symptoms							
EG	43.85 ± 6.28^†^	49.42 ± 10.17	-2.207	.027^∗^	5.57 ± 3.89	-.065	.948
CG	50.28 ± 6.12	54.28 ± 6.72	-2.207	.027^∗^	4.00 ± 0.60		
Systemic symptoms							
EG	19.42 ± 3.45	24.00 ± 4.20	-2.232	.026^∗^	4.58 ± 0.75	-1.236	.217
CG	20.00 ± 5.35	21.57 ± 5.47	-2.032	.042^∗^	1.57 ± 0.12		
Social function							
EG	16.71 ± 5.40	21.42 ± 5.62	-2.214	.027^∗^	4.71 ± 0.22	-.980	.327
CG	17.85 ± 5.72	18.71 ± 4.68	-1.200	.230	0.86 ± 1.04		
Emotional function							
EG	26.57 ± 4.85	29.14 ± 5.49	-2.023	.043^∗^	2.57 ± 0.64	-.265	.791
CG	29.85 ± 6.89	31.71 ± 7.11	-2.121	.034^∗^	1.86 ± 0.22		
Total score							
EG	106.57 ± 13.12	123.85 ± 20.94	-2.226	.026^∗^	17.28 ± 7.82	-1.091	.275
CG	118.00 ± 13.37	126.28 ± 14.67	-2.197	.028^∗^	8.28 ± 1.30		

^†^Mean ± SD. ^∗^*p* < .05. EG: experimental group; CG: control group.

## Data Availability

All required evidence that supports the results of this study has been reported. The other raw data could not be revealed or shared due to ethical concerns and the protection of participants' privacy.
